The article "Effects of Amiodarone and Esmolol for Heart Rate and Cardiovascular Changes" was retracted in 2023. Reasons: signs of a paper mill; suspected computer-generated content; unreliable results or conclusions; lack of ethics approval or compliance.

# Effects of Amiodarone and Esmolol for Heart Rate and Cardiovascular Changes

**DOI:** 10.1155/2022/9197369

**Published:** 2022-06-27

**Authors:** Hao Wang, Fengping Lei, Lei Bai, Anping Zhang

**Affiliations:** ^1^Department of Cardiology, The First People's Hospital of Li County, Longnan 742500, Gansu, China; ^2^Department of Pharmacy, Pharmacy, Xi'an Aerospace General Hospital, Xi'an 710199, Shaanxi, China; ^3^Nursing Department, Children's Hospital of Xi'an Jiaotong University, Xi'an 710002, Shaanxi, China; ^4^Department of Vascular Surgery, Lanzhou University Second Hospital, Lanzhou 730030, Gansu, China

## Abstract

**Objective:**

To probe into the effects of amiodarone and esmolol for heart rate disorders and myocardial infarction.

**Methods:**

76 cases of cardiopathy in our hospital from July 2019 to October 2021 were analyzed for myocardial infarction. The control group applied amiodarone treatment. Blood pressure, treatment effect, adverse reactions, myocardial marker levels, electrocardiogram, and heart function indicators were compared.

**Results:**

There were no statistical differences in two groups of diastolic pressure (*P* > 0.05). The analysis of the systolic pressure in the study group was greater than the control group (*P* < 0.05); The effective rate was higher than that of the control group (*P* < 0.05); the incidence of adverse reactions in the study group and control group was 28.95% and 31.58%, respectively, and there was no statistically significant difference between groups (*P* > 0.05). The standards of markers were significantly reduced compared with the control group (*P* < 0.05). After treatment, the heart rate of the two groups was significantly reduced, and the QT intervals were significantly shortened. But compared with the control group, reduction was larger in the research group (*P* < 0.05). Compared with the control group, the resolution rate was higher (*P* < 0.05). After treatment, the two groups of quality of life were significantly increased, and compared with the control group, the increase in the quality of life of the study group was greater (*P* < 0.05).

**Conclusion:**

Application of amiodarone and esmolol joint treatment can improve the quality of life, improve the level of heart function and myocardial marker, and can reduce Q-T intervals and prognosis. Therefore, amiodarone and esmolol treatment is worth promoting.

## 1. Introduction

Myocardial infarction is a clinically multiexpressive cardiovascular disease. This disease often induces a variety of complications such as arrhythmias, usually in the early stage of myocardial infarction. [1]. In patients with myocardial infarction combined with arrhythmia, the contraction frequency in the room is significantly increased, the corresponding amount of myocardial oxygen is increased, and the symptoms of myocardial necrosis are significantly aggravated. This is the main cause of sudden death and cardiogenic shock in patients [2]. There is a significant decrease in myocardial infarction combined with arrhythmia patients, and it has seriously threatened the safety of patients [3]. Clinical use of amiodarone is effective up to 80%, but because amiodarone has a classic drug loss, there are short absorption, half-life, and individual differences [4]. More and more studies have confirmed that esmolol can also be used in the clinical treatment of patients with myocardial infarction and can be rapidly alleviated by the compression symptoms of the ventricular period, and the early sudden death rate is significantly reduced, which is conducive to the improvement of patient prognosis [5].

The study selected 76 cases of myocardial infarction from July 2019 to October 2021 from our hospital, and the two drugs—amiodarone and esmolol—were used and therapeutic effects and electrocardiogram variations were analysed and reported as follows.

## 2. Data and Methods

### 2.1. General Information

76 cases of of myocardial infarction were chosen from our hospital from July 2019 to October 2021.

#### 2.1.1. Inclusion Criteria

(1) Compliance with arrhythmias and cardiomyopathy; (2) 48 hours of morbidity; (3) treatment compliance height; (4) did not accept other beta-adrenergic receptors to block drugs before the study by the patient.

#### 2.1.2. Exclusion Criteria

(1) Cardiological shock, room transmission block, loss of compensatory heart failure, and (4) malignant tumor. The study group (*N* = 38) included 26 males and 12 females, with an average BMI of 22.57 ± 3.25 kg/m^2^, average disease of 3.12 ± 1.07, and average age of 46.34 ± 2.35 years. The control group (*N* = 38) included 25 males, 13 females, with an average BMI of 22.54 ± 3.24 kg/m^2^, average disease of 3.13 ± 1.05, and an average age of 46.34 ± 2.33 years. This study has been approved by the ethical department. The general data difference between the two groups is statistically significant (*P* > 0.05).

### 2.2. Method

#### 2.2.1. Control Group

5% glucose solution and 20 ml + 3 mg/kg amiodarone injection (national medicine quasi-word H20044923, production enterprise: Shandong Fang Ming Pharmaceutical Group Co., Ltd.) were used, and each intravenous injection time is 10 min. 7 days were required for treatment, and 6 months of prognosis for patients was required.

#### 2.2.2. Study Group

Apply amiodarone treatment based on the treatment of the control group, and the treatment method is the same. Intravenous injection volume is 0.5 mg/(kg·min^−1^) Ezolol (National Medicine Standard H19991059, Production Enterprise: Qilu Pharmaceutical Co., Ltd.), for about 1 min, and the next vein drop control is controlled at 0.05 mg/(kg·min^−1^). After 4 minutes, continue to maintain the dose, and if the effect is not ideal, it can be gradually incremented by 0.05 mg/(kg·min^−1^), but the optimal dose should be controlled at 0.3 mg/(kg·min^−1^). Internally, a total of 7D continuous treatment is received, and the patient was followed up for 6 months prognosis.

## 3. Observation Indicator

### 3.1. Blood Pressure [6]

Blood pressure coupling was used for to patient's blood pressure measurement. Attention should be paid to the patient before the measurement, and patients need to sit still for 5 minutes. The right arm blood pressure was measured by a corrected standard desktop hydraulometer, and the 5th sound of Coriolis is the diastolic pressure. The first sound of Coriolis is the systolic pressure, and the blood pressure is measured. Measurement time interval for each time is 1-2 min, and each blood pressure average is taken as the final value of blood pressure.

### 3.2. Treatment Effect [7]

Nominal symptoms disappear, and electrocardiogram was normal. On further aggravation, the heart rate change is small. Efficiency = (productive + effective) number/total number × 100%.

### 3.3. Adverse Reactions

The incidence of adverse reactions is inversely relative to the prognosis of patients.

### 3.4. Myocardial Marker Level [8]

5 ml of venous blood was drawn and centrifuged at 3000 rpm to obtain serum for N-terminal B-type sodium peptide (NT-probnp), creatine kinase uNP (CK-MB), and myocardial index testing such as hypermorriamalone protein T (HS-TNT). The operation is strictly carried out in accordance with the manufacturer's instructions.

### 3.5. ECG Indicator [9]

### 3.6. Sinus Turpoli Rate

The patients were followed up for 6 months, the sinus rhythm infusion volume was counted, and the transparency rate was calculated to judge the prognosis of patients.

### 3.7. Heart Function Indicators

These include left ventricular ejection fraction (LVEF), left ventricular diastolic volume (LVEDV), and left ventricular shrinkage vector (LVESV) 3 indicators.

### 3.8. Quality Rating [10]

Apply SF-36 meter to assess the patient's social, psychological, emotional, and cognitive functions, forming a total of 100 points. The score is proportional to the quality of life.

### 3.9. Statistical Method

Utilized statistical SPSS22.0 software for data analysis, such as data compliance with normal distribution. Counting data are compared with the comparison ratio and the intergroup differential analysis selection card test. Measurement data (metric ± standard difference) indicate that *P* < 0.05 is statistically significant.

## 4. Results

Two groups of blood pressure comparison between the two sets of diastolic pressure show significant differences (*P* > 0.05) (Table 1).

Two groups of treatment effect contrast control group, the effective rate of the study group was 78.95%, 94.74%, and the research team was efficient than the control group (*P* < 0.05) (Table 2).

The incidence of adverse reactions in two groups was 28.95% and 31.58%, and there was no statistically significant difference in comparison between groups (*P* > 0.05) (Table 3).

After comparison of myocardial markers in two groups, the levels of myocardial markers in the two groups were significantly reduced, but compared with the control group, the research group decreased larger and has statistical significance (*P* < 0.05) (Figure 1).

Two sets of electrocardiogram indicators were compared and showed that the heart rate of two groups was significantly reduced, and the QT intervals were significantly shortened. But compared with the control group, the research group decreased larger and has statistical significance (*P* < 0.05) (Figure 2).

Sinus rhythm removal rate of two groups: compared to the control group, the resolution rate of the group was higher (*P* < 0.05) (Figure 3).

Heart function indicators of two sets were compared to the control group; the LVEDV and LVESV indicators were lower; and the LVEF indicator was higher (*P* < 0.05) (Figure 4).

After the comparison of two groups of quality of life, the two groups of life rating increased significantly, compared with the control group, and the quality of life rating increased larger (*P* < 0.05) (Figure 5).

## 5. Discussion

The data show that the incidence population tends to be young, in which unhealthy lifestyle is the main induced factor [11]. At present, the use of amiodarone treatment can be improved on the symptoms of paroxysmal tachycardia, and it is also suitable for myocardial infarction treatment [12]. Amiodarone is an antiarrhythmic first-line drug, which can block the L-type Ca^2+^, Na^+^, and K^+^ channel, sinus, and junction zone, and the in-room conduction speed is significantly slowed [13]. Another study confirmed that amiodarone will be self-regulatory inhibition of sinus nodules and room interruption; the potential time history is prolonged, which is conducive to the mitigation of ventricular fibrillation and atrial fibrillation; and the clinical treatment is higher [14].

Esmolol is a selective *β*1-receptor blocker. At present, it is increasingly widely used in clinical treatment of cardiopathy with myocardial infarction, and it is of great significance to the improvement of heart function indicators [15]. The QTCD reflects the unevenness of myocardial positivity, but amiodarone is not only used for the transfer but also for sinus regulation. The drug can be extended to the time course of each of the cardiomyoma action potentials and can be excited to return. The process is eliminated, and the speed is significantly slowed [16]. The drug also plays an important role in vascular expansion and improving blood flow. After treatment, the patient's heart rate is significantly reduced [17]. Nevertheless, since the auxiliary of the amiodate is relatively long, the index is large, and it is necessary to reduce the amount of amiodarone in order to reduce the degree of liver function. Esmolol will compete in the binding site of catechine phenol, the function of *β*1-receptor is inhibited, the movement and resting heart rate is slow, and myocardial consumption is significantly reduced [18]. Esmolol is shorter, and it is possible to control atrial fibrillation, which is conducive to ventricular rate control [19]. The study analyzed the influence of the two drugs—esmolol and amiodarone—on patients. The results showed that, after treatment, the two sets of heart rate were significantly reduced, and QT intervals were significantly shortened, but compared with the control group, the research group reduced the magnitude (*P* < 0.05). The results confirmed that amiodarone is safe and effective. Expanding the blood vessels around the coronary artery increased coronary blood flow, and the myocardial oxygen consumption is significantly reduced. In addition, the results showed that the effectiveness of the control group and the study group was 78.95% and 94.74%, and the efficiency of the study group was higher than the control group, but the two groups of adverse reactions were not significantly different. The results confirmed that combined drugs can improve the treatment efficiency, but does not increase adverse reactions, which facilitates the improvement of patient prognosis. And, amiodarone and esmolol have higher safety.

Studies use esmolol treatment, while improving myocardial oxygen consumption, and it can reduce blood pressure. After treatment, the patient's systolic pressure is significantly improved, which is conducive to the clinical symptoms of patients, which can be used as arrhythmia combined with myocardial infarction preferred treatment [20, 21]. Esmolol can reduce the peripheral resistance of coronary artery, which can effectively control the blood volume, while weakening myocardial contraction ability and reducing myocardial infarction, and can improve patient social, psychological, emotional, and cognitive functions. The results showed that, after treatment, the two sets of quality of life were significantly increased, compared with the control group, and the increase in the quality of life of the study group was greater (*P* < 0.05). The results confirmed that amiodarone treatment is conducive to the patient's return to society and can alleviate the negative emotions of patients, and patients can face disease with good attitudes, which is conducive to follow-up treatment and intervention. On the basis of amiodone treatment, the treatment of Esmolol is synergistic, and it is possible to compensate the drug for amiodarone, and it will enhance the drug efficacy [14, 22]. The study showed that, after treatment, the two sets of myocardial markers and cardiac function levels were significantly improved, but the research team improved the improvement. The study was consistent with the study of Liu [23]. However, as arrhythmia is a faster progression, the results will be affected by many factors such as research objects, so subsequent research needs to increase sample quantity and multicenter research and analyze two drugs to prognosis on patients' value and mechanism.

In summary, the use of amiodarone and esmolol in patients with myocardial infarction can improve the quality of life, improve the level of heart function and myocardial marker, and can reduce Q-T intervals and prognosis. Therefore, amiodarone and esmolol treatment is worth promoting [24, 25].

## Figures and Tables

**Figure 1:** Experimental result.

**Figure 2:** Experimental result.

**Figure 3:** Experimental result.

**Figure 4:** Experimental result.

**Figure 5:** Experimental result.

**Table 1:** Two sets of blood pressure contrast (*N*, %).

Group	Count	Shuxo pressure (mmHg)	Sealing pressure (mmHg)
Control group	38	70.47 ± 8.65	103.33 ± 10.51
Research group	38	70.53 ± 10.93	116.83 ± 11.34
*T*	—	1.685	17.524
*P*	—	>0.05	<0.05

**Table 2:** Comparison of two groups of treatment results.

Group	Count	Descendant	Efficient	Invalid	Efficient
Control group	38	20 (52.63)	10 (26.32)	8 (21.05)	78.95%
Research group	38	27 (71.05)	9 (23.68)	2 (5.26)	94.74%
*X* ^2^	—	—	—	—	6.325
*P*	—	—	—	—	<0.05

**Table 3:** Analysis of two groups of preparation.

Group	Count	Liver function injury	Nausea	Sinus arrhythmia	Phlebitis	Hypotension	Incidence
Control group	38	3 (7.89)	2 (5.6)	2 (5.26)	2 (5.26)	2 (5.26)	28.95%
Research group	38	2 (5.26)	3 (7.89)	2 (5.26)	2 (5.26)	3 (7.89)	31.58%
*X* ^2^	—	—	—	—	—	—	6.325
*P*	—	—	—	—	—	—	<0.05

## Data Availability

The raw data supporting the conclusions of this article will be made available by the authors, without undue reservation.
